The article "MiR-22 Inhibition Alleviates Cardiac Dysfunction in Doxorubicin-Induced Cardiomyopathy by Targeting the sirt1/PGC-1α Pathway" was retracted in 2022. Reasons: unreliable results or conclusions; concerns about the images.

# MiR-22 Inhibition Alleviates Cardiac Dysfunction in Doxorubicin-Induced Cardiomyopathy by Targeting the sirt1/PGC-1α Pathway

**DOI:** 10.3389/fphys.2021.646903

**Published:** 2021-04-01

**Authors:** Runze Wang, Yuerong Xu, Xiaolin Niu, Yexian Fang, Dong Guo, Jiangwei Chen, Hanzhao Zhu, Jiaying Dong, Ran Zhao, Ying Wang, Bingchao Qi, Gaotong Ren, Xue Li, Li Liu, Mingming Zhang

**Affiliations:** ^1^Department of Cardiology, Tangdu Hospital, The Fourth Military Medical University, Xi'an, China; ^2^Department of Hematology, Tangdu Hospital, The Fourth Military Medical University, Xi'an, China; ^3^Department of Orthodontics, School of Stomatology, The Fourth Military Medical University, Xi'an, China; ^4^Department of Cardiology, Xijing Hospital, The Fourth Military Medical University, Xi'an, China; ^5^Department of Cardiovascular Surgery, Xijing Hospital, The Fourth Military Medical University, Xi'an, China

**Keywords:** doxorubicin, mitochondrial dysfunction, oxidative stress, mitophagy, miR-22

## Abstract

Doxorubicin (DOX) cardiotoxicity is a life-threatening side effect that leads to a poor prognosis in patients receiving chemotherapy. We investigated the role of miR-22 in doxorubicin-induced cardiomyopathy and the underlying mechanism *in vivo* and *in vitro*. Specifically, we designed loss-of-function and gain-of-function experiments to identify the role of miR-22 in doxorubicin-induced cardiomyopathy. Our data suggested that inhibiting miR-22 alleviated cardiac fibrosis and cardiac dysfunction induced by doxorubicin. In addition, inhibiting miR-22 mitigated mitochondrial dysfunction through the sirt1/PGC-1α pathway. Knocking out miR-22 enhanced mitochondrial biogenesis, as evidenced by increased PGC-1α, TFAM, and NRF-1 expression *in vivo*. Furthermore, knocking out miR-22 rescued mitophagy, which was confirmed by increased expression of PINK1 and parkin and by the colocalization of LC3 and mitochondria. These protective effects were abolished by overexpressing miR-22. In conclusion, miR-22 may represent a new target to alleviate cardiac dysfunction in doxorubicin-induced cardiomyopathy and improve prognosis in patients receiving chemotherapy.

## Introduction

Doxorubicin (DOX) has been a widely used chemotherapy drug since the 1960s, but its widespread use is limited given its dose-dependent cardiotoxicity (Singal and Iliskovic, 1998). In a retrospective study, congestive heart failure (CHF) occurred in 5% of patients who received DOX treatment at a dose of 500–550 mg/m^2^. The incidences of CHF in DOX-treated patients at doses of 551–600 and >601 mg/m^2^ were 16 and 26%, respectively (Swain et al., 2003). Numerous studies have reported that DOX exerts its antineoplastic effect mainly by targeting topoisomerase-II (Top2), damaging DNA (Lyu et al., 2007), and inducing oxidative stress (Zhang et al., 2020), autophagy (Li et al., 2016), and mitochondrial dysfunction (Yin et al., 2018). Hence, it is urgent and vital to identify the underlying mechanism of DOX-induced cardiotoxicity and finally resolve this question.

Mitochondria are the main energy sources of the heart and provide >95% ATP through oxidative phosphorylation (Dorn et al., 2015). Mitochondria are involved in regulating many cellular processes, so normal mitochondrial function is vital for the heart (Hoshino et al., 2013; Lesnefsky et al., 2016; Chistiakov et al., 2018). Mitochondrial homeostasis is the result of mitochondrial biogenesis and the dynamic balance of mitophagy (Picca et al., 2018). Dysregulated mitochondrial biogenesis and mitophagy flux are involved in DOX-induced cardiomyopathy (DOXIC) (Catanzaro et al., 2019; Wallace et al., 2020). Activation of mitochondrial biogenesis mitigated DOXIC mitochondrial dysfunction (Cui et al., 2017). However, the role of mitophagy in DOXIC remains inconsistent. In two different studies, inhibiting mitophagy and activating mitophagy both protected against DOXIC (Yin et al., 2018; Wang, P. et al., 2019).

MicroRNAs (miRNAs) are a class of small single-stranded non-coding RNAs with a length of 19–24 nucleotides that bind to the 3′-untranslated region (3′-UTR) of mRNA, inhibit mRNA translation, and lead to mRNA degradation. It has been reported that miR-22 plays roles in heart diseases, such as diabetic cardiomyopathy, cardiac hypertrophy, and ischemia reperfusion injury, by targeting sirt1 (Huang et al., 2013; Du et al., 2016; Tang et al., 2018). In addition, miR-22 is also involved in DOXIC by targeting sirt1 to regulate oxidative stress (Xu, C. et al., 2020). Although the role of miR-22 in DOXIC has been mentioned, the mechanism of mitochondrial dysfunction remains unclear.

Our study revealed another mechanism of DOXIC in which miR-22 and mitochondrial dysfunction were involved and suggested that miR-22 may be a potential target for DOXIC treatment.

## Methods and Materials

### Transgenic Mice

MiR-22 cardiac-specific knockout (miR-22^cKO^) and miR-22 cardiac-specific overexpression (miR-22^cOE^) mice were generated on the C57BL/6 background and generously provided by Huang Zhanpeng. The genotype of the animals was identified by real-time PCR according to the manufacturer's instructions.

### Cardiotoxicity Induced by Doxorubicin

All experimental mice were approximately 10–12 weeks old. The experimental mice were injected intraperitoneally with doxorubicin at a dose of 5 mg/kg weekly for five consecutive weeks and maintained for 1 week after the last injection (Gupta et al., 2018). The mice were randomly divided into the following groups with *n* = 6 each: 1—(1) wild-type (WT), (2) miR-22^cKO^, (3) DOX, and (4) miR-22^cKO^+DOX; 2—(1) wild-type (WT), (2) miR-22^cOE^, (3) DOX, and (4) miR-22^cOE^+DOX. All experimenters were blind to group assignment and outcome assessment.

### Primary Neonatal Mice Cardiomyocytes Isolation and Culture

The hearts were separated from 1-day-old mice. Atrial tissue was removed, and the mice were washed with PBS to remove blood. Then, ventricular tissues were cut into pieces and digested with 5 ml collagenase type II at a concentration of 1 mg/ml for 7 min. The supernatant was transported into a 15 ml centrifuge tube, and an equal amount of DMEM with 10% fetal bovine serum (FBS) was used to terminate digestion. The above steps were repeated until the tissue was completely digested. The dissociated cells were replated in a culture flask at 37°C for 2 h to enrich the culture with cardiomyocytes. The non-adherent cardiomyocytes were collected and were then plated onto gelatin-coated plates.

### Echocardiography

The experimental animals' cardiac function was measured using an M-mode echocardiography system with a 15 MHz linear transducer (Vevo 2100; Visual Sonics, Toronto, ON, Canada). The left ventricular end-systolic diameter (LVESD) and left ventricular end-diastolic diameter (LVEDD) were measured. The left ventricular ejection fraction (LVEF) and left ventricular fractional shortening (LVFS) were analyzed by computer algorithms (Wang, S. et al., 2019). Each diameter was obtained from five consecutive cardiac cycles and averaged. Data were obtained from three biological repeats.

### Mitochondrial ROS and Total ROS in Primary Cardiomyocytes and Mouse Hearts

Mitochondrial ROS (MitoROS) were detected by using a MitoSOX Red Mitochondrial Superoxide Indicator according to the manufacturer's instructions (Yeasen, Shang Hai). Dihydroethidium (DHE) staining was used to measure cardiac ROS levels as previously described (Hu et al., 2019).

### Western Blotting

Total protein was obtained from the left ventricle tissue. The left ventricle tissue was lysed with RIPA lysis buffer mixed with protease inhibitor cocktail on ice and then homogenized. The complete procedure was described as previous (Zhang et al., 2016). All results were repeated thrice.

### Histological Analysis

A week after the last injection, the hearts were removed, washed with phosphate buffered saline (PBS), and cut into transverse slices through the middle route of the ventricles. Then, the heart slices were fixed in 4% paraformaldehyde overnight, embedded in paraffin, cut into 4 μm thick sections, and stained with Masson's trichrome (Sigma Aldrich, United States). The area of fibrosis was observed in 20 randomly chosen high-power fields (x40) in each section by optical microscopy.

### Wheat Germ Agglutinin (WGA) Staining

Heart samples preparation and wheat germ agglutinin staining (Green, Thermo Fisher Scientific, United States) were performed as previously described (Hu et al., 2019).

### Mitophagy Detected by Fluorescence Imaging

The colocalization of LC3 with mitochondria was used to measure mitophagy. Fluorescence images were obtained using an Olympus FV1000 laser confocal microscope as previously described (Wang, S. et al., 2019).

### Statistical Analysis

All experiment data were analyzed by GraphPad Prism8 software. The results are presented as mean ± SEM. Unpaired 2-tailed Student's *t*-test was performed when comparing two groups, and one-way ANOVA was performed when comparing multiple groups to calculate significance. The results were considered statistically significant when *P* < 0.05.

## Results

### Knocking Out miR-22 Alleviates Cardiac Dysfunction in DOXIC

To identify the function of miR-22 in DOXIC, miR-22 cardiac-specific knockout mice were generated. We first measured cardiac function by echocardiography. One week after the last injection, increased LVEF and LVFS and decreased LVEDD and LVESD were observed in the miR-22^cKO^+DOX group compared to the DOX group, which revealed that knocking out miR-22 alleviated DOXIC cardiac dysfunction (Figures 1A–E). Masson staining suggested an increased fibrotic area in the DOX group compared to the control group, whereas knockout of miR-22 significantly alleviated fibrosis as evidenced by a smaller fibrotic area in the miR-22^cKO^+DOX group compared with the DOX group (Figures 1F,G). In addition, in the miR-22^cKO^+DOX group, DOX-induced cardiac atrophy was mitigated as identified by WGA staining (Figures 1H,I). Finally, decreased serum LDH and CK-MB levels in the miR-22^cKO^+DOX group compared with the DOX group also confirmed that knocking out miR-22 alleviates DOXIC (Figures 1J,K).

**Figure 1:** Knocking out miR-22 alleviates cardiac dysfunction in DOXIC. **(A)** M-mode Echocardiograms representative image (*n* = 6), **(B)** LVEF, **(C)** LVFS, **(D)** LVESD, **(E)** LVEDD, **(F)** Representative images of Masson staining, **(G)** Relative collagen area, **(H)** Representative WGA staining images, **(I)** Relative cell area, **(J)** serum LDH (*n* = 6), **(K)** serum CK-MB (*n* = 6), Data were shown as mean ± SEM. *P < 0.05 vs. saline group, ^‡^*P* < 0.05 vs. DOX group, ^†^*P* < 0.05 vs. miR-22^cKO^ group.

### Knocking Out miR-22 Alleviates Mitochondrial Dysfunction in DOXIC

Mitochondrial dysfunction can cause an increase in reactive oxygen species (ROS). Hence, we detected the level of ROS by DHE staining (Figures 2A,B). DOX treatment caused a significant increase in ROS levels. However, in the miR-22^cKO^+DOX group, the level of ROS was decreased compared with that in the DOX group. Then, western blotting was performed to evaluate mitochondrial biogenesis protein levels in experimental animal hearts. In the DOX group, the levels of PGC-1α, TFAM, and NRF-1 were decreased, whereas protein expression in the miR-22^cKO^+DOX group was increased compared with that in the DOX group (Figures 2C–F). In cardiomyocytes, we measured the level of mitochondrial ROS by a mitoSOX assay kit. In the DOX group, mitoSOX levels were increased, whereas the mitochondrial ROS level decreased when miR-22 was knocked out (Figures 2G,H).

**Figure 2:** Knocking out miR-22 mitigates mitochondrial dysfunction in DOXIC. **(A,B)** Representative images of DHE staining, **(C)** Representative images of blots, **(D)** Relative PGC-1α protein level ratio, **(E)** Relative TFAM protein level ratio, **(F)** Relative NRF-1 protein level ratio, Data were expressed as mean ± SEM. *P < 0.05 vs. saline group, ^‡^*P* < 0.05 vs. DOX group, ^†^*P* < 0.05 vs. miR-22^cKO^ group. **(G,H)** Representative images of mitochondrial ROS in neonatal mice cardiomyocytes, Scale bars = 50 μm. *P < 0.05 vs. NC group, ^‡^*P* < 0.05 vs. NC+DOX group, ^†^*P* < 0.05 vs. miR-22 inhibitor group.

### Knocking Out miR-22 Upregulates Mitophagy in DOXIC

Western blotting results suggested that p62 and LC3-II expression was increased and PINK1 and parkin expression was decreased in the DOX group compared with the Saline group. Moreover, the p62 level of the miR-22^cKO^+DOX group decreased, and the LC3-II level decreased. PINK1 and parkin were increased (Figures 3A–E). It has been reported that sirt1 is one of the targets of miR-22. Hence, we also measured the level of sirt1. As shown in Figure 3F, in the DOX group, the level of sirt1 was decreased compared with that in the Saline group. However, in the miR-22^cKO^+DOX group, sirt1 expression was increased compared with that in the DOX group. *In vitro*, we transfected cardiomyocytes with the dosage of 1 × 10^9^ TU/ml HBAD-GFP-LC3. In the DOX group, the number of LC3 and mitochondrial colocalizations was decreased. In the miR-22 inhibitor+DOX group, the number was increased compared with that in the DOX group (Figures 3G,H). To investigate whether miR-22 exerts its effect by targeting sirt1, we performed a luciferase reporter assay. The results showed that sirt1 was the target of miR-22 (Figure 3I).

**Figure 3:** Knocking out miR-22 improves the level of mitophagy in DOXIC. **(A)** Representative western blots, **(B)** relative p62 protein level ratio, **(C)** LC3II/GAPDH ratio, **(D)** relative PINK1 protein level ratio, **(E)** relative Parkin protein level ratio, **(F)** relative sirt1 protein level ratio, Data were expressed as mean ± SEM. *P < 0.05 vs. saline group, ^‡^*P* < 0.05 vs. DOX group, ^†^*P* < 0.05 vs. miR-22^cKO^ group. **(G)** Representative colocalization images of GFP-LC3 (green) and mitochondria (MitoTracker red), **(H)** Quantitative analysis of GFP-LC3 puncta per cell. *P < 0.05 vs. NC group, ^‡^*P* < 0.05 vs. NC+DOX group, ^†^*P* < 0.05 vs. miR-22 inhibitor group. Scale bars = 2 μm. All the experiments were repeated three times. **(I)** Results of luciferase report. *P < 0.05 vs. NC group in sirt1 group, ^†^*P* < 0.05 vs. NC group in MUT sirt1 group. All the experiments were repeated three times.

### Overexpressing miR-22 Aggravates Cardiac Dysfunction in DOXIC

MiR-22 cardiac-specific overexpressing mice were used to perform gain-of-function experiments. The echocardiography results revealed decreased LVEF and LVFS and increased LVEDD and LVESD in the miR-22^cOE^+DOX group compared with the DOX group, suggesting that overexpressing miR-22 aggravated DOXIC cardiac dysfunction (Figures 4A–E). In addition, overexpressing miR-22 increased the fibrotic area compared with that in the DOX group as evidenced by Masson staining (Figures 4F,G). Moreover, in the miR-22^cOE^+DOX group, DOX-induced cardiac atrophy was aggravated, which was identified by WGA staining (Figures 4H,I). Finally, increased serum LDH and CK-MB levels in the miR-22^cOE^+DOX group compared with the DOX group also demonstrated that overexpressing miR-22 can aggravate DOXIC (Figures 4J,K).

**Figure 4:** Overexpressing miR-22 aggravates cardiac dysfunction in DOXIC. **(A)** M-mode Echocardiograms representative image (*n* = 6), **(B)** LVEF, **(C)** LVFS, **(D)** LVESD, **(E)** LVEDD, **(F)** Representative images of Masson staining, **(G)** Relative collagen area, **(H)** Representative WGA staining images, **(I)** Relative cell area, **(J)** serum LDH (*n* = 6), **(K)** serum CK-MB (*n* = 6), Data were shown as mean ± SEM. *P < 0.05 vs. saline group, ^‡^*P* < 0.05 vs. DOX group, ^†^*P* < 0.05 vs. miR-22^cOE^ group. All the experiments were repeated three times.

### Overexpressing miR-22 Aggravates Mitochondrial Dysfunction in DOXIC

To assess the role of overexpressing miR-22 in DOXIC mitochondrial dysfunction, we performed DHE staining (Figures 5A,B). In the miR-22^cOE^+DOX group, cardiac ROS levels were increased compared with those in the DOX group. Western blot results revealed that mitochondrial biogenesis proteins in experimental animal hearts in the miR-22^cOE^+DOX group were decreased compared with those in the DOX group. PGC-1α, TFAM, and NRF-1 levels were decreased when miR-22 was overexpressed (Figures 5C–F). To investigate whether miR-22 increased the level of mitochondrial ROS, we performed a MitoSOX assay. The data suggested that overexpressing miR-22 increased the level of mitochondrial ROS compared with that in the DOX group (Figures 5G,H).

**Figure 5:** Overexpressing miR-22 aggravates mitochondrial dysfunction in DOXIC. **(A,B)** Representative images of DHE staining, **(C)** Representative images of blots, **(D)** Relative PGC-1α protein level ratio, **(E)** Relative TFAM protein level ratio, **(F)** Relative NRF-1 protein level ratio, Data were expressed as mean ± SEM. *P < 0.05 vs. saline group, ^‡^*P* < 0.05 vs. DOX group, ^†^*P* < 0.05 vs. miR-22^cKO^ group. **(G,H)** Representative images of mitochondrial ROS in neonatal mice cardiomyocytes, Scale bars = 50 μm. *P < 0.05 vs. NC group, ^‡^*P* < 0.05 vs. NC+DOX group, ^†^*P* < 0.05 vs. miR-22 mimic group. All the experiments were repeated three times.

### Overexpressing miR-22 Inhibits Mitophagy in DOXIC

In the miR-22^cOE^+DOX group, western blot results suggested that p62 and LC3-II expression was decreased, and PINK1 and parkin expression was decreased compared with the DOX group (Figures 6A–F). Then, we transfected cardiomyocytes with HBAD-GFP-LC3. In the miR-22 mimic+DOX group, the amount of LC3 localized to mitochondria was decreased compared with that in the DOX group (Figures 6G,H).

**Figure 6:** Overexpressing miR-22 inhibits the level of mitophagy in DOXIC. **(A)** Representative western blots, **(B)** relative p62 protein level ratio, **(C)** LC3II/GAPDH ratio, **(D)** relative PINK1 (PTEN induced putative kinase 1) protein level ratio, **(E)** relative Parkin protein level ratio, **(F)** relative sirt1 protein level ratio, Data were expressed as mean ± SEM. *P < 0.05 vs. saline group, ^‡^*P* < 0.05 vs. DOX group, ^†^*P* < 0.05 vs. miR-22^cOE^ group. **(G)** Representative colocalization images of GFP-LC3 (green) and mitochondria (MitoTracker red), **(H)** Quantitative analysis of GFP-LC3 puncta per cell. Scale bars = 2 μm. *P < 0.05 vs. NC group, ^‡^*P* < 0.05 vs. NC+DOX group, ^†^*P* < 0.05 vs. miR-22 mimic group. All the experiments were repeated three times.

## Discussion

Doxorubicin, a type of cytotoxic chemotherapy drug, exhibits dose-dependent cardiotoxicity. DOX can lead to cardiac atrophy, cardiac fibrosis, and cardiac oxidative stress, which finally causes cardiac dysfunction. Dexrazoxane is the only drug that the Food and Drug Administration (FDA) approved for the treatment of DOX cardiotoxicity (Fang et al., 2019). However, its clinical use has been limited by an increased carcinogenicity risk (Yu et al., 2018). MiRNAs play an important role in DOXIC. Inhibiting miR-23a attenuates DOXIC cardiac dysfunction by targeting the PGC-1α/DRP1 pathway (Du et al., 2019). DOX-induced increased apoptosis and decreased autophagy were improved by miR-146a through the TAF9b/P53 pathway (Pan et al., 2019). Inhibiting miR-451 alleviates cardiac dysfunction by mitigating oxidative stress and reducing apoptosis (Li et al., 2019). MiR-31-5p improved DOXIC dysfunction via quaking and circular RNA Pan3 (Ji et al., 2020).

In addition, numerous studies have confirmed that miR-22 plays an important role in cardiovascular diseases. For example, inhibiting miR-22 can attenuate cardiac hypertrophy by targeting sirt1, whereas upregulating miR-22 contributes to I/R injury by aggravating mitochondrial dysfunction (Huang et al., 2013; Du et al., 2016). In this study, we discovered that inhibiting miR-22 can mitigate DOXIC cardiac dysfunction and that overexpressing miR-22 aggravates DOXIC cardiac dysfunction.

Mitochondria, which provide >90% of ATP for the heart and account for approximately 45% of the volume of cardiomyocytes, play a vital role in DOXIC (Govender et al., 2014). Hence, maintaining good mitochondrial quality control is important for mitochondrial homeostasis. Disrupted mitochondrial biogenesis and enhanced mitochondrial ROS together lead to mitochondrial dysfunction (Zhou et al., 2001). PGC-1α (peroxisome proliferator-activated receptor γ coactivator-1α), a key regulator of mitochondrial biogenesis, and TFAM (mitochondrial transcription factor A), a downstream molecule of PGC-1α, were inhibited in DOXIC, suggesting inhibition of mitochondrial biogenesis in DOXIC (Guo et al., 2014, 2015). Recently, a study suggested that dexmedetomidine attenuated DOXIC via inhibiting mitochondrial ROS production (Yu et al., 2020). Our current study suggested that inhibiting miR-22 activated mitochondrial biogenesis by upregulating PGC-1α, TFAM, and NRF-1. In addition, inhibition of miR-22 also improved cardiac oxidative stress by decreasing ROS levels in the heart and mitochondrial ROS in primary cardiomyocytes. Overexpression of miR-22 aggravated mitochondrial biogenesis inhibition and enhanced oxidative stress.

Mitophagy is a protective process that selectively degrades damaged mitochondria, which is an important process for mitochondrial quality control (Youle and Narendra, 2011; Frank et al., 2012). However, the role of mitophagy in DOXIC remains debatable. Yin et al. revealed that DOX enhanced mitophagy and that inhibiting mitophagy improved DOX-induced cardiac dysfunction (Yin et al., 2018). However, another two studies suggested that DOX inhibited parkin expression, and increased parkin expression can alleviate cardiac dysfunction (Liu et al., 2019; Wang, P. et al., 2019). Most recently, a study revealed that luteolin attenuated DOXIC by enhancing mitophagy (Xu, H. et al., 2020). In our study, DOX treatment inhibited mitophagy, and inhibiting miR-22 rescued mitophagy by increasing PINK1 and parkin expression. Increased LC3 and mitochondrial colocalization was observed in the miR-22 inhibitor+DOX group compared with the DOX group. Promoting mitophagy can alleviate DOX cardiotoxicity. These results provide convincing evidence that mitophagy is a double-edged sword and may play different roles in different stages of disease.

Sirt1 is an NAD^+^-dependent deacetylase that is crucial to mitochondrial biogenesis (Tang, 2016). Studies have reported that sirt1 deacetylates PGC-1α and then regulates mitochondrial biogenesis in various pathological processes (Iwabu et al., 2010; Price et al., 2012; Ding et al., 2018). Recently, a study reported that activating the sirt1/PGC-1α pathway can regulate autophagy/mitophagy and mitigate oxidative stress (Liang et al., 2020). In the current study, our results revealed that enhancing the sirt1/PGC-1α pathway can alleviate DOX-induced mitochondrial dysfunction by increasing mitochondrial biogenesis and mitophagy. It has been reported that sirt1 is one of the targets of miR-22 (Huang et al., 2013). Our results suggest that knocking out miR-22 mitigated DOXIC.

In addition, a study reported that inhibiting miR-22 can decrease oxidative stress (Xu, C. et al., 2020). Our data also identified that knocking out miR-22 reduces ROS levels in the heart and decreases mitochondrial ROS in cardiomyocytes. In conclusion, our current study revealed that miR-22 targets the sirt1/PGC-1α pathway to regulate mitochondrial biogenesis and mitophagy and then to alleviate mitochondrial dysfunction. MiR-22 may represent a new potential target for DOXIC treatment.

## Limitation

Other signaling pathways may have participated in the link between miR-22 and its effects in DOXIC. The function of cardiomyocytes is closely related to mitochondria biogenesis, and mitochondrial dysfunction is a primary cause of DOXIC. To further demonstrate the efficacy of miR-22 administration on mitochondrial biogenesis and function, mitochondria fusion and fission related pathway should be measured in future studies. Further studies are needed to investigate whether miR-22 exerts its effects by different mechanisms in DOXIC mice.

## Data Availability Statement

The raw data supporting the conclusions of this article will be made available by the authors, without undue reservation.

## Ethics Statement

The animal study was reviewed and approved by Care and Use of Laboratory Animals and the Guidelines for the Welfare of Experimental Animals issued by the Ethics Committee on Animal Care of the Fourth Military Medical University.

## Author Contributions

MZ, XL, and LL defined the topic of this project and revised the manuscript carefully. RW, YX, XN, and YF performed the laboratory experiments and wrote the manuscript. JC, HZ, YW, RZ, DG, BQ, GR, and JD analyzed the data. MZ translated literature and polished the manuscript. RW and YX established the animal model. All authors carried out the work, read, and approved the final manuscript.

## Conflict of Interest

The authors declare that the research was conducted in the absence of any commercial or financial relationships that could be construed as a potential conflict of interest.
